The article "Speckle Tracking Algorithm-Based Ultrasonic Cardiogram in Evaluation of the Efficacy of Dexmedetomidine Combined with Bundle Strategy on Patients with Severe Sepsis" was retracted in 2023. Reasons: signs of a paper mill; suspected computer-generated content; unreliable results or conclusions; concerns about the data.

# Speckle Tracking Algorithm-Based Ultrasonic Cardiogram in Evaluation of the Efficacy of Dexmedetomidine Combined with Bundle Strategy on Patients with Severe Sepsis

**DOI:** 10.1155/2021/7179632

**Published:** 2021-10-25

**Authors:** Chang'an Lv, Guan Wang, Aidong Chen

**Affiliations:** ^1^Department of Critical Care Medicine, Affiliated Hospital of Jiangnan University, Wuxi 214062, China; ^2^Hospitalization Management Section, Affiliated Hongqi Hospital of Mudanjiang Medical University, Mudanjiang 157011, China; ^3^Digestive Department, Affiliated Hongqi Hospital of Mudanjiang Medical University, Mudanjiang 157011, China

## Abstract

The research aimed to study the effect of dexmedetomidine combined with bundle strategy on the cardiac function of patients with severe sepsis through pyramid speckle tracking algorithm-based echocardiography, expected to provide reference for its clinical treatment. 98 patients with severe sepsis or septic shock admitted to the hospital were selected as the research subjects, and they were equally divided into experimental group (dexmedetomidine + bundle strategy) and control group (dexmedetomidine + routine nursing), with 49 in each. Ultrasonic cardiogram examination was performed on patients before and after treatment, and the pyramid-based speckle tracking (PST) algorithm was designed and used. The results showed that the running time of the PST algorithm (105.25 s) was less than that of the BM algorithm (336.41 s), and the difference was statistically significant (*P* < 0.05), and the systolic blood pressure, diastolic blood pressure, left ventricular wall, and heart rate of the experimental group before treatment were not significantly different from those of the control group (*P* > 0.05). The ultrasound index results found that the ejection fraction (EF) and fractional shortening (FS) of the two groups of patients showed a downward trend over time (1–7 days), while the *E*/*A* ratio showed an upward trend, and the *E*/*A* ratio of the experimental group was significantly greater than the control group (*P* < 0.05). The systolic blood pressure, diastolic blood pressure, left ventricular wall, and heart rate of the two groups of patients showed a downward trend over time (1–7 days), and the systolic blood pressure, diastolic blood pressure, left ventricular wall, and heart rate of the experimental group were significantly lower than those of the control group (*P* < 0.05). The 28-day mechanical ventilation time (6.97 ± 3.11 days), intensive care unit (ICU) stay time (9.18 ± 2.86 days), and the 28-day mortality rate (15.31%) of the experimental group were lower than those of the control group (6.97 ± 3.11 days; 13.08 ± 2.53 days; 31.95%) (*P* < 0.05). In conclusion, the PST algorithm can effectively improve the quality of echocardiography and assist physicians in clinical evaluation, and dexmedetomidine combined with bundle strategy can stabilize the heart rate and reduce myocardial oxygen consumption in severe sepsis, while effectively shortens the recovery time and improves the overall prognosis.

The article "Speckle Tracking Algorithm-Based Ultrasonic Cardiogram in Evaluation of the Efficacy of Dexmedetomidine Combined with Bundle Strategy on Patients with Severe Sepsis" was retracted in 2023. Reasons: signs of a paper mill; suspected computer-generated content; unreliable results or conclusions; concerns about the data.

## 1. Introduction

Sepsis is a disorder of the body's response caused by infectious factors, leading to organ dysfunction. It is a common complication of severe trauma, major surgery, and infection and is also one of the most common causes of death in critically ill patients [1, 2]. Big data shows that more than 19 million people worldwide suffer from sepsis each year, of which approximately 6 million patients die due to ineffective treatment, and the mortality rate is as high as 25%. Worse still, nearly 3 million survivors develop cognitive dysfunction [3–5]. Patients with sepsis usually have symptoms such as fever (body temperature > 38.5°C), chills (body temperature < 36°C), accelerated heart rate (heart rate > 90 beats/min), rapid breathing (respiratory rate > 20 beats/min), and decreased urination. The conventional clinical treatment for patients with septic shock is still to use fluid resuscitation and positive muscle support to re-establish organ and tissue perfusion and oxygen delivery. Although this method can alleviate the low effective circulating blood volume and the hypotension, it fails to improve the compliance and diastolic function of ventricular muscle [6].

With the accumulation of experience in the treatment of sepsis, in addition to antibiotics and glucocorticoids, sedation and analgesia are found to be instrumental in reducing the release of inflammatory factors and inhibiting excessive activation of neuroendocrine, and dexmedetomidine, a new highly selective adrenal gland receptor agonist, has become a good choice [7, 8]. Despite much research on the treatment of sepsis with different concentrations of dexmedetomidine, its effects on the myocardial perfusion and cardiac function of septic patients remain to be verified [9]. Bundled nursing treatment refers to the collection of evidence-based treatments and nursing measures to deal with an intractable disease, and each intervention in the group of measures is clinically proven to improve patient outcomes. In this study, dexmedetomidine and bundle strategy were used to treat patients with severe sepsis in order to provide new ideas for the treatment of sepsis.

Medical ultrasound can display the structure of the body, such as tendons, muscles, joints, blood vessels, and internal organs, so as to help doctors find the source of the disease. The diagnostic imaging for heart-related diseases is called ultrasonic cardiogram [10, 11]. Nowadays, the ultrasonic cardiogram has been routinely used in the diagnosis of any suspected or known heart disease patients, and it can provide a lot of useful information, including the size and shape of the heart, pumping capacity, and the location and scope of any tissue damage. In addition, combining mathematical models with imaging can also improve clinical diagnosis. Ultrasound speckles specifically correspond to internal tissue of the human body, which reflects the movement of the tissues to a certain extent [12]. The echo intensity of the speckle area is stronger versus the nonspeckle area. In the ultrasound image, it manifests as brighter speckle area darkness around the speckle area. Speckle tracking technology uses the best pattern matching technology to track and identify the spatial movement of echo speckles in the myocardium based on high-frame two-dimensional gray-scale ultrasound images and track its position in each frame of the image. It is a new quantification method to evaluate the torsional deformation of the heart. Hence, on the basis of image segmentation, researcher can extract and track the speckles [13].

The article "Speckle Tracking Algorithm-Based Ultrasonic Cardiogram in Evaluation of the Efficacy of Dexmedetomidine Combined with Bundle Strategy on Patients with Severe Sepsis" was retracted in 2023. Reasons: signs of a paper mill; suspected computer-generated content; unreliable results or conclusions; concerns about the data.

Above, in this study, 98 patients with severe sepsis or septic shock were randomly divided into experimental groups (dexmedetomidine + bundle strategy) and control group (dexmedetomidine + routine nursing). They all had the ultrasonic cardiogram examination before and after treatment, and a pyramid-based speckle tracking (PST) algorithm was designed, expected to provide reference for the clinical care and treatment of patients with severe sepsis.

## 2. Materials and Methods

### 2.1. Research Subjects

In this study, 98 patients with severe sepsis or septic shock who were admitted to the Hospital from March 10, 2019, to April 25, 2021, were selected as research subjects, including 56 males and 42 females, aged 30–65 years old. According to different treatment plans, they were equally divided into experimental group (dexmedetomidine + bundle strategy) and control group (dexmedetomidine + routine nursing). This study has been approved by the Medical Ethics Committee of Hospital. The patients and their families understood this study and signed the informed consent.

Inclusion criteria are as follows: (1) all patients had normal sinus rhythm; (2) all patients had good treatment compliance; (3) all patients had normal systolic blood pressure; and (4) all were under 18 years old. Exclusion criteria are as follows: (1) patients with severe cardiac insufficiency; (2) patients with coronary heart disease; (3) patients with moderate to severe mitral regurgitation; (4) patients with end-stage malignant tumors; (5) patients with severe liver and kidney dysfunction; and (6) patients whose sequential organ failure assessment (SOFA) [14] scores were greater than 2 points.

The article "Speckle Tracking Algorithm-Based Ultrasonic Cardiogram in Evaluation of the Efficacy of Dexmedetomidine Combined with Bundle Strategy on Patients with Severe Sepsis" was retracted in 2023. Reasons: signs of a paper mill; suspected computer-generated content; unreliable results or conclusions; concerns about the data.

### 2.2. Treatment Plan

Patients in the control group were treated with dexmedetomidine combined with routine nursing. First, routine nursing was given, including intravenous rehydration and Wanhan injection for fluid resuscitation, and the patient's central venous pressure was increased to 8 cm H_2_O. After that, a micropump was used to inject dexmedetomidine at 5 *μ*g/kg/h for 10 minutes.

Patients in the experimental group were treated with dexmedetomidine combined with bundle strategy. First, bundled nursing was given. (1) The central venous pressure and central venous blood oxygen saturation were monitored within 3 hours. (2) For those who did not respond to fluid resuscitation within 6 hours, hypertensive drugs were used to maintain the patient's average arterial pressure at ≥65 mmHg. For those with an increased lactic acid level, they were re-examined, aimed to restore the lactic acid level to the normal. (3) After fluid resuscitation, a micropump was used to inject dexmedetomidine at 5 *μ*g/kg/h for 10 minutes. (4) Psychological care for patients: it was necessary to understand the main complaints of patients and communicate with them to improve their enthusiasm and compliance.

Observation indicators are as follows: the SOFA score and acute physiology and chronic health (APACHE-II) score at 1, 3, 5, and 7 days after treatment and the mechanical ventilation time, intensive care unit (ICU) stay, and 28-day mortality.

### 2.3. Ultrasonic Cardiogram Examination

The patients were scanned with the V-3000 phased array ultrasound diagnosis system from the United States of America. With the two-chamber view of the patient's apex as the measurement plane, the filter was set to a low level, and the gain was adjusted properly. The sampling line was parallel to the anterior wall of the left ventricle, and 5 periodic spectra were stored on the CD for analysis. The indexes to be measured included the factional shortening (FS) and the ratio of early mitral valve blood flow velocity (*E*) to peak mitral valve filling velocity (*A*) during atrial contraction (*E*/*A* ratio). At the same time, the left ventricular wall thickness was measured, and the ejection fraction (EF) was calculated.

### 2.4. PST Algorithm

The PST algorithm combines the image pyramid method and the block matching method. It can be used to calculate the similarity of two image blocks. Its operating principle is shown in Figure 1. A pyramid model is built based on the module block and the block to be matched, and the absolute error sum is calculated [15]. Then, each pixel in the search window is searched, and the similarity from the top to the bottom was analyzed. Finally, the result is output. This algorithm can effectively reduce the traditional absolute error and the workload of the algorithm.  Figure 2 shows the pyramid model.

The article "Speckle Tracking Algorithm-Based Ultrasonic Cardiogram in Evaluation of the Efficacy of Dexmedetomidine Combined with Bundle Strategy on Patients with Severe Sepsis" was retracted in 2023. Reasons: signs of a paper mill; suspected computer-generated content; unreliable results or conclusions; concerns about the data.

Figure 2 is a pyramid model. The size of the model is 2^5^ × 2^5^ pixels, and the pixel value of the upper layer is equal to the sum of the pixel values of the adjacent lower layer. The pyramid is expressed as follows:

(1) $$\begin{array}{c} W^{t-1}\left(i,j\right)=W^{t}\left(2i-1,2j-1\right)+W^{t}\left(2i-1,2j\right)+W^{t}\left(2i,2j-1\right)+W^{t}\left(2i,2j\right), \end{array}$$

where *W*^*t*^(*i*, *j*) represents the pixel value of the position (*i*, *j*) in the *t*th layer of the pyramid. During transportation, the absolute error sum is calculated as follows:

(2) $$\begin{array}{c} S_{\mathrm{total}}=\sum_{i=1}^{2^{t}}\sum_{j=1}^{2^{t}}\left|W^{t}\left(i,j\right)-Q^{t}\left(i,j\right)\right|, \end{array}$$

where *S*_total_ represents the absolute error sum, *W*^*t*^ represents the original image block, and *Q*^*t*^ represents the image block to be tested. Then, the following equation is obtained after further analysis:

(3) $$\begin{array}{c} S_{\mathrm{total}}=\sum_{i=1}^{2^{t}}\sum_{j=1}^{2^{t}}\left\{\begin{array}{c} \left|W^{t}\left(2i-1,2j-1\right)-Q^{t}\left(2i-1,2j-1\right)\right|+\left|W^{t}\left(2i-1,2j\right)-Q^{t}\left(2i-1,2j\right)\right|\\ +\left|W^{t}\left(2i,2j-1\right)-Q^{t}\left(2i,2j-1\right)\right|++\left|W^{t}\left(2i,2j\right)-Q^{t}\left(2i,2j\right)\right| \end{array}\right\}. \end{array}$$

Then, Minkowski's inequality [16] was introduced, and equation (3) can be converted to the following equation:

(4) $$\begin{array}{c} S_{\mathrm{total}}\geq \left|\sum_{i=1}^{2^{t}}\sum_{j=1}^{2^{t}}W^{t}\left(i,j\right)\right|-\left|\sum_{i=1}^{2^{t}}\sum_{j=1}^{2^{t}}Q^{t}\left(i,j\right)\right|. \end{array}$$

Hence, for a module of 2^*t*^ × 2^*t*^, there are

(5) $$\begin{array}{c} S_{\text{total}}^{t}\left(i,j\right)\geq S_{\text{total}}^{t-1}\left(i,j\right). \end{array}$$

Equation (5) is then expanded to get the following equation:

(6) $$\begin{array}{c} S_{\mathrm{total}}^{t}\left(i,j\right)\geq S_{\mathrm{total}}^{t-1}\left(i,j\right)\geq S_{\mathrm{total}}^{t-2}\left(i,j\right)\geq S_{\mathrm{total}}^{t-3}\left(i,j\right)\geq \cdots \geq S_{\mathrm{total}}^{0}\left(i,j\right). \end{array}$$

This top-down similarity measurement method can effectively reduce the running time. In terms of complexity, the algorithm mainly involves addition, subtraction, multiplication, and absolute value operations. With a module of 64 × 64 as an example, the construction of pixels in a 7-layer pyramid requires 3 operations, and the total number of operations is as follows:

(7) $$\begin{array}{c} \mathrm{times}=3\times \sum_{l=1}^{6}2^{l-1}\times 2^{l+1}. \end{array}$$

Then, for a *T*-level pyramid, the computational amount of the algorithm is expressed as follows:

(8) $$\begin{array}{c} \mathrm{time}s^{T}=\sum_{l=0}^{T}\left(3\times 2^{2n}-1\right). \end{array}$$

Figure 3 shows the addition, subtraction, and absolute value of a 64 × 64 module. Obviously, the amount of computation increases rapidly from top to bottom.

The article "Speckle Tracking Algorithm-Based Ultrasonic Cardiogram in Evaluation of the Efficacy of Dexmedetomidine Combined with Bundle Strategy on Patients with Severe Sepsis" was retracted in 2023. Reasons: signs of a paper mill; suspected computer-generated content; unreliable results or conclusions; concerns about the data.

### 2.5. Statistics

The data were processed by SPSS19.0, the measurement data were expressed by the mean ± standard deviation ($\bar{x}\pm s$), and the count data were expressed by a percentage (%). One-way analysis of variance was used for pairwise comparison. *P* < 0.05 was the threshold for significance.

## 3. Results

### 3.1. Basic Information of Subjects

Figure 4 shows the basic data of the two groups of patients. It was noted that the differences in age, sex ratio, SOFA score, and APACHE-II score between the experimental group and the control group were not statistically significant (*P* > 0.05).

### 3.2. Simulation Analysis of Algorithm Performance

With the left ventricle video as an example, a 16-pixel translation is performed on each frame in the video, and the search window size was 16, and the image block size was 17. The PST algorithm in this study was compared with the traditional block matching (BM) algorithm for the operation accuracy and operation time [17].

Figure 5 shows the operating accuracy and operation time of the PST algorithm and the BM algorithm. It was noted that the accuracy of the PST algorithm (97.05%) was not statistically significant (*P* > 0.05) compared with that of the BM algorithm (95.33%), while the running time of the PST algorithm (105.25 s) was less than that of the BM algorithm (336.41 s), and the difference was statistically significant (*P* < 0.05).

Figure 6 shows the running volume of each layer of the pyramid. The algorithm operates from the top to the bottom. At the top layer, the absolute error sum of the 248 pixels was calculated. On the 0th layer, the ratio of the pixels that met the conditions was 94.76%, and the ratio decreased layer by layer. On the 4th layer, the ratio was only 8.87%. In addition, the amount of calculation increased as the number of layers increased. The number of operations for a single pixel increased from 2 on the 0th layer to 749 on the fourth layer, and the total number of operations increased from 496 on the 0th layer to 16478 on the fourth layer.

The article "Speckle Tracking Algorithm-Based Ultrasonic Cardiogram in Evaluation of the Efficacy of Dexmedetomidine Combined with Bundle Strategy on Patients with Severe Sepsis" was retracted in 2023. Reasons: signs of a paper mill; suspected computer-generated content; unreliable results or conclusions; concerns about the data.

### 3.3. The Segmentation Effects of Different Algorithms on the Ultrasonic Cardiogram

Figure 7(a) is an ultrasonic cardiogram of a 45-year-old female patient with no history of palpitation, shortness of breath, and chest pain. It was noted that the variability of the inferior vena cava was 10%, the right heart was not enlarged, and systolic and diastolic functions of the left ventricle were reduced. The blue smooth and closed contour line in Figure 7(b) is the contour of the left ventricle. The speckles around the contour line were tracked to obtain the movement of the speckles (Figure 7(c)). It was noted that the movement of the speckles was periodic, in line with the basic operating law of the heart.

Figure 8(a) is an ultrasonic cardiogram of a 60-year-old male patient who complained of fever and general fatigue, with a history of schizophrenia, benign prostatic hyperplasia, hypertension, and long-term indwelling catheterization. The blue smooth and closed contour line in Figure 8(b) is the contour of the left ventricle. The speckles around the contour line were tracked to obtain the movement of the speckles (Figure 8(c)). It was noted that the movement of the speckles was periodic, in line with the basic operating law of the heart.

### 3.4. Comparison of Cardiac Function before Treatment

Figure 9 shows the cardiac function between the two groups of patients before treatment. It was noted that the differences in systolic blood pressure, diastolic blood pressure, left ventricular wall, and heart rate were not statistically significant between the experimental group and the control group (*P* > 0.05).

### 3.5. Comparison of Ultrasound Indexes between the Two Groups of Patients before and after Treatment

Figure 10 shows the ultrasound indexes between the two groups of patients before and after treatment. It was noted that the EF and FS of the two groups of patients showed a downward trend over time (1–7 days), while the *E*/*A* ratio showed an upward trend. The EF and FS of the experimental group were not statistically different from those of the control group (*P* > 0.05). In addition, the *E*/*A* ratio of the experimental group was significantly greater than that of the control group, and the difference was statistically significant (*P* < 0.05).

### 3.6. Cardiac Function Indexes of the Two Groups of Patients after Treatment

Figure 11 shows the cardiac function indexes of the two groups of patients after treatment. It was noted that the systolic blood pressure, diastolic blood pressure, left ventricular wall, and heart rate of the two groups of patients showed a downward trend over time (1–7 days). The systolic blood pressure, diastolic blood pressure, left ventricular wall, and heart rate of the experimental group were significantly lower than those of the control group, and the difference was statistically significant (*P* < 0.05).

The article "Speckle Tracking Algorithm-Based Ultrasonic Cardiogram in Evaluation of the Efficacy of Dexmedetomidine Combined with Bundle Strategy on Patients with Severe Sepsis" was retracted in 2023. Reasons: signs of a paper mill; suspected computer-generated content; unreliable results or conclusions; concerns about the data.

### 3.7. Comparison of Mechanical Ventilation Time, ICU Stay, and 28-Day Mortality Rate between the Two Groups

Figure 12 shows the mechanical ventilation time, ICU stay, and 28-day mortality rate of the two groups of patients. It was noted that the 28-day mechanical ventilation time (6.97 ± 3.11 days), ICU stay time (9.18 ± 2.86 days), and the 28-day mortality rate (15.31%) of the experimental group were lower than those of the control group (6.97 ± 3.11 days; 13.08 ± 2.53 days; 31.95%) (*P* < 0.05).

## 4. Discussion

Studies have confirmed that the excessive activation of neuroendocrine in the early stage of sepsis and the large release of inflammatory factors are important causes of cardiac dysfunction and myocardial damage. Therefore, in recent years, *α*2 adrenergic receptor agonists have received extensive attention [18]. Dexmedetomidine can be used as an *α*2 adrenergic receptor agonist in the treatment of sepsis, which can regulate the body fluid of peripheral tissue [19]. Bundle strategy for sepsis treatment emphasizes the importance of completing diagnosis and treatment measures within a certain period of time. It standardizes and streamlines the monitoring and treatment of sepsis so to identify the condition as early as possible. In this study, the bundle strategy and dexmedetomidine were used to optimize the clinical treatment plan. First, the PST algorithm was constructed, and it was found that the operating accuracy of the PST algorithm was not statistically significant compared with the BM algorithm (*P* < 0.05), and the operation time of the PST algorithm was significantly shorter than that of the BM algorithm, and the difference was statistically significant (*P* < 0.05), which was in line with the results of Berge et al. [20], indicating that the PST algorithm can optimize the operation process and shorten the operation time. As for the segmentation effects of the ultrasonic cardiogram, the movement of speckles selected by the PST algorithm was periodic, consistent with the basic operating law of the heart [21].

98 patients with severe sepsis or septic shock were equally divided into experimental group (dexmedetomidine + bundle strategy) and control group (dexmedetomidine + routine nursing). In the experimental group, the systolic blood pressure, diastolic blood pressure, left ventricular wall, and heart rate before treatment were not statistically different from those of the control group (*P* > 0.05), ensuring the feasibility of subsequent studies [22, 23]. Then, the ultrasound indexes of the two groups of patients before and after treatment were compared. It was found that the EF and FS of the two groups of patients showed a downward trend over time (1–7 days), while the *E*/*A* ratio showed an upward trend. The EF and FS of the experimental group were not statistically significant compared with those of the control group (*P* > 0.05). In addition, the *E*/*A* ratio of the experimental group was significantly greater than that of the control group, and the difference was statistically significant (*P* < 0.05). Hence, the *E*/*A* ratio based on the PST algorithm can effectively reflect the patient's curative effects [24]. The systolic blood pressure, diastolic blood pressure, left ventricular wall, and heart rate of the two groups of patients showed a downward trend over time (1–7 days). The systolic blood pressure, diastolic blood pressure, left ventricular wall, and heart rate of the experimental group were significantly lower than those of the control group (*P* < 0.05). It suggested that dexmedetomidine + bundle strategy can stabilize the heart rate and reduce myocardial oxygen consumption and improve the systolic and diastolic function of patients [25]. In the experimental group, the mechanical ventilation time and ICU stay were shorter and the 28-day mortality rate was lower versus the control group, and the difference was statistically significant (*P* < 0.05). It can be inferred that dexmedetomidine combined with bundle strategy can effectively shorten the recovery time and improve the overall prognosis [26].

The article "Speckle Tracking Algorithm-Based Ultrasonic Cardiogram in Evaluation of the Efficacy of Dexmedetomidine Combined with Bundle Strategy on Patients with Severe Sepsis" was retracted in 2023. Reasons: signs of a paper mill; suspected computer-generated content; unreliable results or conclusions; concerns about the data.

## 5. Conclusion

In this study, 98 patients with severe sepsis or septic shock were divided into experimental group (dexmedetomidine + cluster care) and control group (dexmedetomidine + routine nursing). They all had the ultrasonic cardiogram examination before and after treatment, and the PST algorithm was used. The results found that the constructed algorithm in this study is better than the traditional algorithm, which can effectively improve the quality of echocardiography, and dexmedetomidine combined with bundle strategy can stabilize the heart rate and reduce myocardial oxygen consumption in severe sepsis, while effectively shortening the recovery time required and improving the overall prognosis. However, in the study, a 65-year-old patient experienced a sharp drop in heart rate and blood pressure, which required the help of vasoactive drugs to stabilize the circulation. Although it was excluded from the experimental group, it also suggested that dexmedetomide should be used with caution in elderly patients. The safe dose is still to be confirmed by more clinical trials. However, some limitations in the study should be noted. The sample size is small, which will reduce the power of the study. In the follow-up, an expanded sample size is necessary to strengthen the findings of the study. In conclusion, the results of this study provide reference for the clinical care and treatment of patients with severe sepsis.

The article "Speckle Tracking Algorithm-Based Ultrasonic Cardiogram in Evaluation of the Efficacy of Dexmedetomidine Combined with Bundle Strategy on Patients with Severe Sepsis" was retracted in 2023. Reasons: signs of a paper mill; suspected computer-generated content; unreliable results or conclusions; concerns about the data.

## Figures and Tables

**Figure 1:** Flowchart of the PST algorithm.

**Figure 2:** The pyramid model.

**Figure 3:** Calculation amount of the algorithm: (a) addition; (b) subtraction; (c) absolute value.

**Figure 4:** Basic information of the subjects: (a) the age and sex ratio; (b) the SOFA score and APACHE-II score.

**Figure 5:** Operating accuracy and operation time of the PST algorithm and BM algorithm. *Note*. ^*∗*^ means significant difference compared with the PST algorithm (*P* < 0.05).

**Figure 6:** The segmentation effects of the three algorithms on CT angiography: (a) the number of pixels; (b) the ratio of pixels that met the conditions; (c) the number of operations for a single pixel; (d) the total number of operations.

**Figure 7:** Ultrasonic cardiogram of a 45-year-old female patient: (a) the original ultrasonic cardiogram; (b) the left ventricular segmentation diagram; (c) the left ventricular movement displacement diagram.

**Figure 8:** Ultrasonic cardiogram of a 60-year-old male patient: (a) the original ultrasonic cardiogram; (b) the left ventricular segmentation diagram; (c) the left ventricular movement displacement diagram.

**Figure 9:** Comparison of cardiac function between the two groups of patients before treatment: (a) the patient's systolic and diastolic blood pressure; (b) the patient's left ventricular wall and heart rate.

**Figure 10:** Comparison of ultrasound indexes between the two groups before and after treatment: (a) EF; (b) FS; (c) *E*/*A* ratio. *Note*. ^*∗*^ indicates that the difference was statistically significant compared with the experimental group (*P* < 0.05).

**Figure 11:** Cardiac function indexes of the two groups of patients after treatment: (a) systolic blood pressure; (b) diastolic blood pressure; (c) left ventricular wall; (d) heart rate. *Note*. ^*∗*^ indicates that the difference was statistically significant compared with the experimental group (*P* < 0.05).

**Figure 12:** Comparison of the duration of mechanical ventilation, length of ICU stay, and 28-day mortality rate between the two groups. Note: (a) 1: the patient's 28-day mechanical ventilation time; 2: the ICU stay time; (b) the patient's 28-day mortality rate; ^*∗*^ indicates that the difference was statistically significant compared with the experimental group (*P* < 0.05).

The article "Speckle Tracking Algorithm-Based Ultrasonic Cardiogram in Evaluation of the Efficacy of Dexmedetomidine Combined with Bundle Strategy on Patients with Severe Sepsis" was retracted in 2023. Reasons: signs of a paper mill; suspected computer-generated content; unreliable results or conclusions; concerns about the data.

## Data Availability

The data used to support the findings of this study are available from the corresponding author upon request.
